The article "The PI3K/mTOR dual inhibitor NVP‐BEZ235 stimulates mutant p53 degradation to exert anti‐tumor effects on triple‐negative breast cancer cells" was retracted in 2026. Reasons: duplicated images; unreliable data; unreliable results or conclusions.

# The PI3K/mTOR dual inhibitor NVP‐BEZ235 stimulates mutant p53 degradation to exert anti‐tumor effects on triple‐negative breast cancer cells

**DOI:** 10.1002/2211-5463.12806

**Published:** 2020-03-06

**Authors:** Jiajing Cai, Jingruo Xia, Jiang Zou, Qiang Wang, Qiang Ma, Ru Sun, Hebin Liao, Lei Xu, Dongsheng Wang, Xiaolan Guo

**Affiliations:** ^1^ Department of Laboratory Medicine Affiliated Hospital of North Sichuan Medical College Nanchong China; ^2^ Department of Laboratory Medicine North Sichuan Medical College Nanchong China; ^3^ Translational Medicine Research Center North Sichuan Medical College Nanchong China

**Keywords:** autophagy, mechanistic target of rapamycin signal transduction pathway, mutant p53, NVP‐BEZ235, protein kinase B, triple‐negative breast cancer

## Abstract

Nearly half of human cancers harbor p53 mutations, and mutant p53 (mutp53) promotes carcinogenesis, metastasis, tumor recurrence and chemoresistance. mutp53 is observed in 30% of breast carcinomas, including triple‐negative breast cancer (TNBC), and thus mutp53 is a promising target for treatment of TNBC. In this study, we investigated the effect of a phosphatidylinositide 3 kinase/mammalian target of rapamycin dual inhibitor, NVP‐BEZ235 (BEZ235), on two TNBC cell lines with mutp53: MDA‐MB‐231 and MDA‐MB‐468. Cell growth, migration and colony‐formation abilities were detected by 3‐(4,5‐dimethylthiazol‐2‐yl)‐2,5‐diphenyl‐tetrazolium bromide, scratch assay, transwell and soft agar assay, revealing that BEZ235 can inhibit the growth, migration and colony‐formation abilities of TNBC cells. In addition, BEZ235 caused degradation of mutp53 in these cells. We investigated the underlying mechanism by inhibiting proteasome function using MG132 and inhibiting autophagy using 3‐methyladenine and shRNAs. We observed that BEZ235 may induce autophagy through repression of the Akt/mammalian target of rapamycin signaling pathway. The observed interplay between mutp53 and autophagy in TNBC cells was examined further by knockdown of ATG5 and ATG7, revealing that degradation of mutp53 induced by BEZ235 may be independent of the ubiquitin–proteasome pathway and autophagy mediated by ATG5 and ATG7. Moreover, we found evidence of positive feedback between mutp53 and autophagy in TNBC cells. In conclusion, BEZ235 may exert antitumor effects against TNBC cells by targeting mutp53, and this may have implications for the development of future therapies.

## Graphical abstract

NVP‐BEZ235 is a phosphatidylinositide 3 kinase/mammalian target of rapamycin dual inhibitor, which exerts an antitumor effect against two triple‐negative breast cancer cell lines harboring mutant p53 protein: MDA‐MB‐231 and MDA‐MB‐468. BEZ235 induces autophagy in these cells, possibly through repression of the AKT/mammalian target of rapamycin pathway. Degradation of mutant p53 induced by BEZ235 is independent of the ubiquitin–proteasome pathway and autophagy. BEZ235 may be a potential therapeutic target for triple‐negative breast cancers with mutant p53.

The article "The PI3K/mTOR dual inhibitor NVP‐BEZ235 stimulates mutant p53 degradation to exert anti‐tumor effects on triple‐negative breast cancer cells" was retracted in 2026. Reasons: duplicated images; unreliable data; unreliable results or conclusions.

**Abbreviations**
AMPK: AMP‐activated protein kinase
BC: breast cancer
DMEM: Dulbecco's modified Eagle's medium
GAPDH: glyceraldehyde‐3 phosphate dehydrogenase
mTOR: mammalian target of rapamycin
MTT: 3‐(4,5‐dimethylthiazol‐2‐yl)‐2,5‐diphenyl‐tetrazolium bromide
mutp53: mutant p53
p‐: phosphorylated
PI3K: phosphatidylinositide 3 kinase
TNBC: triple‐negative breast cancer

Breast cancer (BC) is the most frequent cancer among women. Triple‐negative breast cancer (TNBC) that does not express the estrogen receptor, progesterone receptor and human epidermal growth factor receptor‐2 accounts for approximately 15–25% of BCs 1. Because TNBCs are very easy to metastasize and confer chemoresistance, the current standard therapies for TNBCs are neoadjuvant chemotherapy and radiotherapy. Although early TNBCs have higher response to neoadjuvant chemotherapy, the advanced TNBCs show poor clinical prognosis. TNBCs lack a standard care approach guided by tumor biology 2.

Tumor suppressor protein p53 (TP53) can protect cells from malignant transformation as a cellular guardian. However, as the most commonly mutated gene in human cancers, mutant p53 (mutp53) not only loses tumor suppressor function but gains oncogenic functions 3. Because about 30% of BCs and more than 80% of basal‐like BCs harboring mutp53 genes 4, and TNBCs overlap with basal‐like BC, targeting mutp53 may represent a promising approach for the treatment of TNBCs 5.

As a dual inhibitor of phosphatidylinositide 3 kinase (PI3K)/mammalian target of rapamycin (mTOR), NVP‐BEZ235 (called BEZ235 thereafter) could exert antitumor effects and induce cancer cell apoptosis in multiple trials 6, 7. PI3K and the downstream molecules AKT and mTOR compose the PI3K/AKT/mTOR signaling pathway to regulate cell growth, survival and metabolism in physiological and pathological conditions. Plenty of studies have confirmed that the antitumor effect of BEZ235 was related to the inhibited PI3K/AKT/mTOR pathway. Meanwhile, the systemic antitumor effect of BEZ235 with other conventional chemotherapeutic agents on several cancer cells has been verified 8, 9. However, its effect on TNBC cells was rarely reported.

In this study, we intend to confirm the antitumor effect of BEZ235 on TNBC cells and explore the possible mechanisms more than the inhibited Akt/mTOR pathway, hoping to provide a novel therapeutic approach to treat BCs harboring mutp53.

The article "The PI3K/mTOR dual inhibitor NVP‐BEZ235 stimulates mutant p53 degradation to exert anti‐tumor effects on triple‐negative breast cancer cells" was retracted in 2026. Reasons: duplicated images; unreliable data; unreliable results or conclusions.

## Materials and methods

### Cells and reagents

Human TNBC cell lines MDA‐MB‐231 (p53R280K), MDA‐MB‐468 (p53R273H) and MDA‐MB‐157 (p53 null) were obtained from the Department of Laboratory Medicine, Chongqing Medical University (China, Chongqing). MDA‐MB‐231 was maintained in Dulbecco's modified Eagle's medium (DMEM), whereas MDA‐MB‐468 and MDA‐MB‐157 were grown in Leibovitz's L‐15 (L15) supplemented with 10% fetal bovine serum (HyClone; GE Healthcare Life Sciences, Logan, UT, USA), penicillin (100 U·mL^−1^) and streptomycin (100 μg·mL^−1^; Sigma‐Aldrich; Merck KGaA, Darmstadt, Germany). Cells were incubated in a humidified incubator under 5% CO_2_ at 37 °C. NVP‐BEZ235 was purchased from LC Laboratories (Woburn, MA, USA), and MG‐132 and 3‐methyladenine (3‐MA) were purchased from Sigma‐Aldrich (Merck KGaA). All primary antibodies, including P53 (#2524), LC3 (#4108), phosphorylated (p)‐Akt (#9271), p‐mTOR (#2971), p‐P70S6K (#9205), p‐AMP‐activated protein kinase (p‐AMPK; #2535), p‐MDM2 (#3521), Akt (#4685), mTOR (#2983), P70S6K (#2708), p‐AMPK (#5832), p‐MDM2 (#86934) and glyceraldehyde‐3 phosphate dehydrogenase (GAPDH; #2118) were obtained from Cell Signaling Technology (Beverly, MA, USA).

### MTT viability assay

Cells were seeded in a 96‐well plate (2 × 10^3^ per well) and incubated for 24 h. BEZ235 was added to each well in a concentration series and incubated for 12, 24 and 36 h, respectively. Twenty microliters of 3‐(4,5‐dimethylthiazol‐2‐yl)‐2,5‐diphenyl‐tetrazolium bromide (MTT; 5 mg·mL^−1^; Sigma‐Aldrich) was added to each well and incubated for 4 h at 37 °C, 100 μL DMSO was added to each well and the plate was agitated for 10 min. Absorbance was detected at 490 nm by a multimode detection platform (Molecular Devices Austria GmbH, Wals, Austria). Inhibition rate was calculated as: [(A control − A blank) − (A treated − A blank)]/(A control − A blank) × 100.

### Scratch assay

Cells were seeded in a six‐well plate (5 × 10^5^ cells/well) and cultured until a confluent monolayer was formed. A 10‐μL pipette tip was used to create a scratch. Then the medium was removed and the cells were washed with PBS to clear the nonadherent cells. MDA‐MB‐231 was treated with 2 μm BEZ235, and MDA‐MB‐468 was treated with 0.2 μm BEZ235. The cell migration ability was checked by the closure of the scratch, observed at 24 and 60 h after incubation, respectively. Images were obtained by an inverted microscope (CKX41; Olympus, Tokyo, Japan).

### Transwell migration assay

Cells suspended in DMEM or L15 medium containing 5% FBS were seeded in the upper chamber (6 × 10^4^) of transwell inserts (Corning Incorporated, Corning, NY, USA) with or without BEZ235. MDA‐MB‐231 was treated with 2 μm BEZ235, and MDA‐MB‐468 was treated with 0.2 μm BEZ235. DMEM or L15 supplemented with 20% FBS was added to the lower chamber as an attractant solution. After 72‐h incubation, the remaining cells on the upper chamber were cleared, and the cells that had migrated to the underside of the chamber were fixed by methanol and stained with Giemsa. The migration ability was checked by the number of cells that had migrated to the underside of the chamber. Images were photographed by an inverted microscope.

The article "The PI3K/mTOR dual inhibitor NVP‐BEZ235 stimulates mutant p53 degradation to exert anti‐tumor effects on triple‐negative breast cancer cells" was retracted in 2026. Reasons: duplicated images; unreliable data; unreliable results or conclusions.

### Soft agar assay

Cells (8 × 10^3^) suspended in DMEM or L15 medium containing 0.6% soft agar were seeded in a 60‐mm dish precoated with 3.0% agar in complete growth medium and cultured in a 5% CO_2_ humidified atmosphere at 37 °C. MDA‐MB‐231 was treated with 2 μm BEZ235, and MDA‐MB‐468 was treated with 0.2 μm BEZ235. The medium was replaced every 4 days. After incubation for 16 days, colonies were photographed by an inverted microscope.

### Quantitative RT‐PCR

Total RNA was isolated by TRIzol (Invitrogen, Carlsbad, CA, USA), and cDNA was synthesized from 2 μg RNA by PrimeScript™ Reverse Transcriptase (Takara Bio, Shiga, Japan). The quantitative PCR was conducted with SYBR^®^ Premix Ex Taq^™^ II (Takara Bio) and the LightCycler^®^ 480 System (Roche, Basel, Switzerland) according to the manufacturer's protocol. The primer sequences used for quantitative PCR analysis were as follows: p53, forward 5′‐CCAGGGCAGCTACGGTTTC‐3′ and reverse 5′‐CTCCGTCATGTGCTGTGACTG‐3′; GAPDH, forward 5′‐GCAAGCAGGAGTATGACGAG‐3′ and reverse 5′‐CAAATAAAGCCATGCCAATC‐3′. The relative expressions of all genes were quantified using $2^{-\Delta \Delta C_{t}}$ method. GAPDH was used as internal control.

### Western blot

Cell lysates were extracted with lysis buffer, and protein concentrations were measured by bicinchoninic acid method. An equal amount of proteins was subjected to SDS/PAGE and transferred to poly(vinylidene difluoride) membrane electrophoretically. After blocking, the membranes were incubated overnight with primary antibodies at 4 °C and incubated with proper secondary antibodies for 1 h at room temperature. At last, the protein signals were detected by Fusion FX7 (VILBER, Paris, France).

### shRNA transfection

Transfection mix was prepared according to the manufacturer's instructions (Invitrogen) and added to HEK293T for 48‐h incubation. The supernatant of the HEK293T was collected to treat TNBC cells. Selection antibiotic at the killing concentration was added to TNBC cells until all the cells in the killing control plate are dead. At last, the rest of the cells were collected to validate the stable expression of protein of interest via western blot.

The article "The PI3K/mTOR dual inhibitor NVP‐BEZ235 stimulates mutant p53 degradation to exert anti‐tumor effects on triple‐negative breast cancer cells" was retracted in 2026. Reasons: duplicated images; unreliable data; unreliable results or conclusions.

### Plasmids

pLKO.1 lentiviral plasmids containing shRNAs against ATG5 (TRCN000000150645) and ATG7 (TRCN0000007584) were obtained from Sigma‐Aldrich (Mission shRNA). shp53 pLKO.1 puro (Addgene plasmid 19119), pCMV‐Neo‐Bam p53‐R273H (Addgene plasmid 16439) and pCMV‐Neo‐Bam p53‐R175H (Addgene plasmid 16436) were purchased from Addgene (Cambridge, MA, USA).

### Statistical analysis

graphpad prism 5 (GraphPad Software Inc., San Diego, CA, USA) was used for statistical analysis. Data were expressed as mean ± SD. Student's *t*‐test and one‐way ANOVA test were performed for data comparison. A *P*‐value <0.05 was considered statistically significant.

## Results

### BEZ235 could inhibit the proliferation, migration and colony‐formation abilities of TNBC cells

To determine the antitumor effect of BEZ235 on TNBC cells (MDA‐MB‐231 and MDA‐MB‐468), we treated cells with different concentrations of BEZ235. According to the results of the MTT, BEZ235 suppressed the proliferation of TNBC cells in a time‐ and dose‐dependent manner (Fig. 1A). The scratch assay indicated that BEZ235 could inhibit the migration of TNBC cells (Fig. 1B), and the same result was obtained from the transwell assay (Fig. 1C). The colony‐formation ability of TNBC cells was evaluated by soft agar assay, and the results showed that the number and size of colonies were reduced on BEZ235 exposure compared with the control group (Fig. 1D).

**Figure 1:** BEZ235 could inhibit the proliferation, migration and colony‐formation abilities of TNBC cells. (A) The cell proliferation was detected by MTT assay, displaying the dose‐ and time‐dependent effect of BEZ235 treatment on TNBC cells. The inhibited effect of BEZ235 on cell migration was illustrated by scratch assay (B). Scale bar, 100 μm. (C) Transwell assay was also performed to check cell migration. Scale bar, 50 μm. (D) The colony‐formation ability of TNBC cells was evaluated by soft agar assay. Scale bar, 200 μm. The error bars indicate the standard deviation. The *P* value was calculated using Student's *t*‐test. These results are representative of at least three independent replicates. *P < 0.05. BEZ, BEZ235; CON, control.

### The Akt/mTOR signaling pathway was related to the autophagy induced by BEZ235

To elucidate the mechanisms of the antitumor effect of BEZ235 on TNBC cells, we detected the expressions of key proteins in the Akt/mTOR pathway that play an important role in stimulating cell growth and proliferation, and also relate with autophagy. Akt and mTOR, which are the autophagic negative regulatory factors, were decreased on BEZ235 exposure. Meanwhile, p70S6K, which acts as the cell translation regulation factor, was also down‐regulated after BEZ235 treatment (Fig. 2A). In addition, we observed that BEZ235 initiated autophagy in TNBC cells by the increased LC3, which is the commonly used autophagy marker. Meanwhile, AMPK was enhanced, which could promote autophagy under glucose starvation 10 (Fig. 2B). These results demonstrated that the autophagy initiated by BEZ235 could be related to the suppression of the Akt/mTOR pathway.

The article "The PI3K/mTOR dual inhibitor NVP‐BEZ235 stimulates mutant p53 degradation to exert anti‐tumor effects on triple‐negative breast cancer cells" was retracted in 2026. Reasons: duplicated images; unreliable data; unreliable results or conclusions.

**Figure 2:** The Akt/mTOR signaling pathway was related to the autophagy induced by BEZ235. TNBC cells were treated with an indicated concentration of BEZ235 for 24 h; the total and phosphorylated protein of Akt, mTOR and p70 were analyzed by western blot (A), as well as AMPK and LC3 (B). GAPDH was used as a loading control. The error bars indicate the standard deviation. The *P* value was calculated using Student's *t*‐test. These results are representative of at least three independent replicates. *P < 0.05.

### BEZ235 degraded mutp53 in TNBC cells

In addition to the suppressed Akt/mTOR pathway, we found that BEZ235 also degraded mutp53 by western blot (Fig. 3A). Meanwhile, we checked the p53 mRNA expression of TNBC cells after BEZ235 treatment. The results showed that the p53 mRNA in MDA‐MB‐231 cells was decreased gradually with the exposure time, whereas it did not down‐regulate significantly until upon BEZ235 exposure for 36 h in MDA‐MB‐468 cells (Fig. 3B). Because mutp53 could exert the opposite effects of wtp53 to stimulate the proliferation and migration of cancer cells, especially TNBC cells 11, 12, we hypothesized the antitumor effect of BEZ235 might be related with mutp53 inhibition and the Akt/mTOR pathway repression.

**Figure 3:** BEZ235 degraded mutp53 in TNBC cells. (A) The expressions of P53 and MDM2 were analyzed by western blot after the indicated concentration of BEZ235 for 24‐h treatment. (B) The mRNA expression of p53 was detected by quantitative PCR when TNBC cells were treated with BEZ235 for 24 and 36 h, respectively. GAPDH was used as a loading control. The error bars indicate the standard deviation. The *P* value was calculated using Student's *t*‐test and one‐way ANOVA test. These results are representative of at least three independent replicates. *P < 0.05.

### The mutp53 degradation mediated by BEZ235 was independent with the ubiquitin–proteasome pathway and autophagy

P53 degradation is related to the ubiquitin–proteasome pathway. MDM2, the E3 ubiquitin ligase, acts as the negative regulator of p53 by mediating the degradation of p53 protein and inhibiting the transcriptional activity of p53 13. We confirmed that MDM2 was inhibited by BEZ235 (Fig. 3A), and mutp53 was still decreased after BEZ235 treatment even though the activity of proteasome was inhibited by MG132 (Fig. 4A). Therefore, we hypothesized that the p53 degradation induced by BEZ235 might not relate to the ubiquitin–proteasome pathway. Beyond that, numerous studies have confirmed that autophagy is an intricate, conserved process that could degrade damaged organelles and unfolded proteins; then we speculated that BEZ235 might degrade mutp53 through autophagy. However, BEZ235 also degraded mutp53 after autophagy was suppressed by 3‐MA and shRNAs embedding ATG5/ATG7, respectively (Fig. 4B,C). In conclusion, the p53 degradation initiated by BEZ235 was independent with the ubiquitin–proteasome pathway and autophagy mediated by ATG5 and ATG7.

The article "The PI3K/mTOR dual inhibitor NVP‐BEZ235 stimulates mutant p53 degradation to exert anti‐tumor effects on triple‐negative breast cancer cells" was retracted in 2026. Reasons: duplicated images; unreliable data; unreliable results or conclusions.

**Figure 4:** The mutp53 degradation mediated by BEZ235 was independent with ubiquitin–proteasome pathway and autophagy. (A) After MG132 exposure (10 μm for 4 h), TNBC cells were treated with BEZ235, and P53 expression was assessed. (B) The inhibition effect of 3‐MA and shRNAs embedding ATG5/ATG7. (C) P53 expression was detected on BEZ235 exposure after autophagy was inhibited by 3‐MA, shATG5 and shATG7, respectively. GAPDH was used as a loading control. The error bars indicate the standard deviation. The *P* value was calculated using Student's *t*‐test and one‐way ANOVA test. These results are representative of at least three independent replicates. *P < 0.05.

### There was mutual regulation between mutp53 and autophagy in TNBC cells

More and more studies have indicated the interplay between p53 and autophagy is intertwined and intricate 14, 15. In our study, we found the expressions of LC3 and p‐AMPK were inhibited after mutp53 was suppressed by shRNA in MDA‐MB‐231 and MDA‐MB‐468 cells (Fig. 5A), and these two proteins were increased after the overexpression of mutp53 (R273H/R175H) in MDA‐MB‐157 (p53 null) cells (Fig. 5B). These results indicated that mutp53 might promote autophagy in TNBC cells. Meanwhile, we found that p53 was down‐regulated in MDA‐MB‐231 and MDA‐MB‐468 cells after autophagy was inhibited by shRNAs against ATG5 or ATG7 (Fig. 5C). Based on the earlier results, we concluded that there was positive feedback between mutp53 and autophagy in TNBC cells.

**Figure 5:** There was mutual regulation between mutp53 and autophagy in TNBC cells. The expressions of LC3 and p‐AMPK were detected after p53 was suppressed by shRNA in TNBC cells (A) and the overexpression of mutp53 (R273H/R175H) in MDA‐MB‐157 (p53 null) (B). (C) P53 was measured in TNBC cells after autophagy was inhibited by shRNAs embedding ATG5 and ATG7, respectively. GAPDH was used as a loading control. The error bars indicate the standard deviation. The *P* value was calculated using Student's *t*‐test and one‐way ANOVA test. These results are representative of at least three independent replicates. *P < 0.05.

The article "The PI3K/mTOR dual inhibitor NVP‐BEZ235 stimulates mutant p53 degradation to exert anti‐tumor effects on triple‐negative breast cancer cells" was retracted in 2026. Reasons: duplicated images; unreliable data; unreliable results or conclusions.

## Discussion

We confirmed BEZ235 could suppress the proliferation, migration and colony conformation abilities of TNBC cells in a time‐ and dose‐dependent manner. Not only were mTOR and Akt down‐regulated, but the downstream target p70 was suppressed after BEZ235 treatment. The antitumor effect of BEZ235 on TNBC cells was related to the suppressed Akt/mTOR pathway. In addition, autophagy was induced on BEZ235 exposure that is an intricate, conserved process that plays controversial roles in tumorigenesis and tumor development 16. Autophagy is accelerated by AMPK, which is an important energy sensor and modulates cellular metabolism to maintain energy homeostasis 17. Under glucose starvation, AMPK accelerates autophagy by activating Ulk1 via phosphorylation of Ser317 and Ser777. On the contrary, autophagy is inhibited by mTOR. Under nutrient sufficiency, mTOR prevents Ulk1 activation by phosphorylating Ulk1 Ser757 and disrupting the interaction between Ulk1 and AMPK 18. Accordingly, we speculated BEZ235 could exert an antitumor effect on TNBC cells by inhibiting the Akt/mTOR pathway, and the suppressed mTOR would promote autophagy to affect its antitumor effect.

In our study, we observed the down‐regulation of mutp53 after BEZ235 treatment in TNBC cells for the first time. mutp53 loses the tumor suppressor function and contributes to cancer development and progression through gain of functions such as transcriptional repression and activation, coaggregation with other tumor suppressors and so on. Targeting mutp53 may represent a novel therapeutic for cancer treatment; therefore, mutp53 degradation would contribute to the antitumor effect of BEZ235.

P53 is tightly modulated by posttranslational modification and proteasomal degradation through MDM2. The activation of the PI3K/Akt pathway results in phosphorylation of MDM2 on Ser166 and Ser186, which is necessary for the entrance of MDM2 to the nucleus 19; MDM2 attaches ubiquitin to target p53 for proteasomal degradation 20. From our results, MDM2 was suppressed after BEZ235 treatment, so we speculated that the mutp53 degradation induced by BEZ235 might not relate to the proteasomal degradation, and we confirmed this speculation by using the proteasome inhibitor MG132. The results showed that BEZ235 still decreased mutp53 after MG132 pretreatment. Meanwhile, some research has indicated autophagy was responsible for mutp53 degradation during restriction of glucose; inhibiting autophagy by chemical inhibitors or suppressing autophagic genes would result in mutp53 stabilization, and overexpression of these genes could lead to mutp53 degradation 21, 22, 23, 24, 25. In our research, autophagy inhibitor 3‐MA and shRNAs embedding ATG5/ATG7 were applied to inhibit autophagy, respectively, but mutp53 was still decreased by BEZ235; these results indicated the mutp53 degradation initiated by BEZ235 might not relate to autophagy. In summary, the BEZ235‐induced mutp53 degradation might not relate to ubiquitin–proteasome degradation and the autophagy mediated by ATG5 and ATG7, which could be modulated by posttranscription and other modifications.

The article "The PI3K/mTOR dual inhibitor NVP‐BEZ235 stimulates mutant p53 degradation to exert anti‐tumor effects on triple‐negative breast cancer cells" was retracted in 2026. Reasons: duplicated images; unreliable data; unreliable results or conclusions.

More importantly, we explored the interplay between mutp53 and autophagy. The dual role of p53 in regulating autophagy depends on its subcellular localization. Nucleus p53 can activate AMPK and suppress mTOR to trigger autophagy; it also transactivates plenty of pro‐autophagic genes, including *DRAM*, *ARF* and *DAPK‐1*. Although cytoplasmic p53 may suppress the extranuclear pro‐autophagic function of smARF and interfere with Atg17 to inhibit autophagy 26, 27, different mutp53 variants may play different roles in the regulation of autophagy. mutp53‐R273L and mutp53‐R273H, which preferentially localized in cytoplasm, could inhibit autophagy, whereas mutp53‐R282W and mutp53‐P151H, which preferentially localized in the nucleus, fail to counteract autophagy 28. In addition, mutp53 suppresses autophagy by various mechanisms. Most importantly, mutp53 could inhibit AMPK through their direct interaction or by the inhibition of Sestrins' expression 29. Second, mutp53 could activate the Akt/mTOR pathway and repress the ULK1/Beclin‐1 axis, which is needed to facilitate the initial steps of autophagy 29. Meanwhile, the mutp53/p50 complex could inhibit ATG12 gene promoter and lead to the blockage of autophagy 30. Some authors also reported that mutp53‐R175H, mutp53‐R248W and mutp53‐R273H might increase intracellular reactive oxygen species and lead to the stabilization of HIF‐1α, which can inhibit autophagy in cancers 28. Finally, several mutp53 genes could lead to the induction of mitochondrial citrate carrier, which is pivotal to maintain mitochondrial homeostasis and inhibit autophagic cell death 29. On the contrary, p53 is thought to promote autophagy via activating the transcription of autophagy‐related genes, such as *Dram* and *Isg20L1* 14. Overall, the precise mechanisms by which p53 regulates autophagy are complicated and remain to be determined.

However, there is very little research focus on how autophagy regulates p53. White 14 has indicated that autophagy could suppress p53 by inhibiting AMPK and oxidative stress, which could activate p53, and autophagy could refrain p53 activation by providing substrates for DNA replication and repair. Meanwhile, p53 can be degraded by chaperone‐mediated autophagy 22, 31. Our findings showed there was a positive feedback between mutp53 and autophagy in TNBC cells. We speculated that different mutp53 variants and their various subcellular localizations would play different roles in the modulation of autophagy and the dual role of autophagy in the initiation and development of cancer; even the cell type might affect the regulation between p53 and autophagy.

The article "The PI3K/mTOR dual inhibitor NVP‐BEZ235 stimulates mutant p53 degradation to exert anti‐tumor effects on triple‐negative breast cancer cells" was retracted in 2026. Reasons: duplicated images; unreliable data; unreliable results or conclusions.

In conclusion, our research has suggested that BEZ235 could inhibit the proliferation, metastasis and colony‐conformation abilities of TNBC cells via targeting mutp53; it may have therapeutic benefits for patients with cancer who are carrying mutp53. In addition, the precise interplay between mutp53 and autophagy needs to be deeply investigated, because modulating their interaction would contribute to the treatment for patients with cancer in the future.

## Conflict of interest

The authors declare no conflict of interest.

## Author contributions

DW and XG were involved in the conception of the article and designed the article. JC, JX, JZ and QW collected and assembled the data. QM and RS performed the data analysis and interpretation of the article. HL and LX were involved in the provision of study materials. DW and XG performed the critical revision of the manuscript. JC wrote the manuscript. All authors approved the final version of the manuscript.
